# Analysis of the Evolution of Time and Space Differences and Coordinated Development Degree of Tourism Economy Based on Regional Internet of Things Technology

**DOI:** 10.1155/2021/4415989

**Published:** 2021-11-30

**Authors:** Su Zhang

**Affiliations:** Tourism College of Zhejiang, Hangzhou, Zhejiang 311231, China

## Abstract

From the time dimension, this paper analyzes the characteristics of the scale, industrial structure, employment flexibility, and comprehensive employment effects of regional tourism employment based on the three-level criteria of the scope of tourism employment based on the regional Internet of Things. From the spatial dimension, we take the regional city as the basic research unit, adopt multiple indicators, and conduct a comprehensive evaluation of the regional development of regional tourism employment through horizontal and vertical comparisons. This paper uses multiple linear regression analysis to establish the relationship between the development level of the county tourism economy and the influencing factors; in order of magnitude of influence, they are tourism resource endowment, location traffic conditions, and economic development. Using a combination of a single indicator and multiple indicators, the county tourism economy is evaluated and analyzed for differences in time and space. We select the total tourism revenue as an indicator and use methods such as range, standard deviation, coefficient of variation, and coefficient to analyze the time difference of the tourism economy in each county. We adopt the Granger causality test and other methods to analyze the factors affecting tourism employment in the area and the growth mode. Through the establishment of a structural model of the tourism employment growth dynamics system, causality test and other methods are adopted to analyze the regional tourism employment influencing factors and growth methods, and the results show that the regional tourism employment growth mode is an investment-driven tourism employment growth mode.

## 1. Introduction

In recent years, the development speed of the tourism industry based on the regional Internet of Things has been accelerating, and the level of development has also been increasing. Compared with other regions, especially the developed tourism regions, there is still a relatively large gap, and the overall development level is still relatively low [1]. The travel rate can reflect the number of tourists and tourism income in a region, as well as the tourism development status of a region. There are obvious temporal and spatial differences in the travel rate of cities and states in the same area [2]. In addition to the improvement of people's living standards and scientific and cultural quality, tourism has become a sunrise industry for regional economic and social development [3]. The development of the tourism industry has greatly increased regional national income and effectively increased the gross national product and fiscal revenue; the tourism industry has a relatively large degree of relevance and a strong development driving effect, which can promote the development of related industries and the economy and promote structural optimization and adjustment [4]. The tourism industry is a labor-intensive industry that can accommodate and absorb more labor, create abundant employment space, and help solve social employment problems; the development of the tourism industry improves the quality of life of the people. Not only it can improve people's physical and mental health but also can improve people's quality and accomplishment and enrich people's spiritual world, promote the all-round development of people, and help build a harmonious society [5].

Domestic research studies on the spatial and temporal distribution characteristics of tourism flows have more research on the spatial distribution of inbound tourism flows [6]. Talari et al. [7] divided the regional inbound tourism flow into spatial divisions. For the research on the spatial pattern of tourism flow, in the horizontal pedigree, more emphasis is placed on the study of the circle structure, and in the vertical pedigree, more emphasis is placed on the single-point level study [8]. At present, the conceptual models of the spatial structure of tourism flow mainly include leisure vacation mode, travel mode, spatial layered movement mode, international tourism flow mode, urban tourism flow mode, and tourist travel spatial structure mode [9]. Piccialli and Chianese [10] conducted a research on the theory of tourism flow spatial pattern and divided the basic theory of tourism flow spatial pattern into three theories, namely, circle structure theory, core edge theory, and spatial diffusion theory. And on this basis, some problems existing in the study of tourism flow are put forward. Perles et al. [11] studied the spatial structure optimization of the regional outbound tourism flow and optimized it from the two aspects of the destination and the source of tourists by studying the characteristics of the regional outbound tourism flow and its spatial structure. Foreign scholars have mainly studied tourists' travel preferences, travel motives, travel behavior, travel demand, and the analysis and prediction of travel flows [12]. Zsarnoczky [13] analyzed five factors that directly affect the bilateral flow of tourism flows, namely, political factors, economic factors, private enterprises, intangible factors, and diplomatic and health factors. Weber et al. [14] emphasized the seasonality of tourism flows. From a macroperspective, it uses register-based data to analyze the spatial structure and analyzes the recent impact of tourist flow and migration flows and the flow of foreign property ownership. Jha et al. [15] carried out research on the comparative advantages of tourism flows. The article pointed out that tourism and international trade flows have similarities. The results are usually supported by two aspects: supply-side variables and the comparative advantages of exporting countries. In addition, western geographers are also committed to the study of the interpretation mode and spatial distribution mode of tourism flow, but they are mostly based on hypotheses, so they are of little practical significance, and they have made useful contributions to the research methods of tourism flow [16]. Some scholars analyzed five factors that directly affect the bilateral flow of tourism flows, namely, political factors, economic factors, private enterprises, intangible factors, and diplomatic and health factors [17]. Researchers emphasize the seasonality of tourism flows [18]. An article pointed out that tourism and international trade flows have similarities, and the results are usually supported by two aspects: supply-side variables and the comparative advantage of exporting countries [19]. In addition, Western geographers are also committed to the study of interpretation models and spatial distribution models of tourism flows, but most of them are based on assumptions, which are of little practical significance and have not made useful contributions to the research methods of tourism flows. The study of tourism flow is an important basis for formulating tourism development plans, determining source markets, and formulating external publicity strategies [20, 21].

At present, the research on the difference of tourism economy based on the regional Internet of Things is slightly insufficient. The existing research results are limited to large regions or intercity areas, and most of them are still qualitative analysis, lacking quantitative empirical analysis. This article uses quantitative, qualitative, and spatial analysis methods to study the spatial and temporal differences of the tourism economy based on the regional Internet of Things, analyzes the influencing factors of the differences, and then proposes countermeasures for the development of the county tourism economy on this basis. In view of the characteristics of the temporal and spatial differences in the travel rate, the reasons for these characteristics are analyzed from the aspects of politics, society, tourism resources, transportation, and short-term crises. This method of calculating how much labor input is needed to reverse the output of the tourism industry believes that the employment capacity of tourism characteristic industries mainly depends on two major factors. Based on the actual situation, suggestions are made to increase the travel rate and promote the sustainable development of the regional tourism industry: establish the concept of grand tourism and innovate the concept of tourism development, which is conducive to accelerating the system reform; strengthening the government's leadership in the tourism industry is conducive to regional tourism; focusing on the training of tourism professionals is conducive to improving the quality of tourism services.

## 2. Construction of a Model for the Evolution of Temporal and Spatial Differences in Tourism Economy Based on the Regional Internet of Things Technology

### 2.1. Regional IoT Spatial Hierarchy

In a type of real-time system such as the Internet of Things, Time Computation Tree Logic (TCTL) can represent a large number of naturally occurring normative attributes, such as security and time response, and is especially suitable for research on time reachability. Because of its powerful functions, it can capture many routine inspections and can perform verification more effectively. Since the state space of the underlying model is basically uncountable, the analysis of accessibility must use symbolic technology to describe the continuity of the clock through a finite quotient.  Figure 1 shows the spatial hierarchical nesting of regional IoT.

Due to the real-time and concurrent characteristics of the Internet of Things system, based on exhaustive search for multiplying the state space and the clock band, the number of states generated tends to increase exponentially, which greatly increases time and space consumption. When the number of concurrent systems is large, searching the state space directly will exceed the memory limit of the computer, and the verification result will not be obtained.

(1) $$\begin{array}{c} p\left(x\left(1\right),x\left(2\right),\ldots ,x\left(n\right)\right)=\prod_{i=1}^{n}p\left[x\left(n\right)|x\left(n-i+1\right)\right],\\ C=2\times \frac{{\left(p\left(x\right)\times p\left(n\right)\right)}^{1/2}}{\left(p\left(x\right)+p\left(n\right)\right)}. \end{array}$$

The direct consumption coefficient, also called the input coefficient, is recorded as *i*, *j*, which refers to the direct consumption of the unit's total output of the *j* product (or industry) sector in the production and operation process. The value of the goods or services consumed in the *i* product sector is represented by the direct consumption coefficient of each product (or industry) sector in the form of a direct consumption coefficient table or a direct consumption coefficient matrix, usually represented by the letter *T*.

(2) $$\begin{array}{c} f\left(x\right)=x\left(i\right)+\frac{x\left(i\right)\times x\left(j\right)}{x\left(i\right)+x\left(j\right)},\\ T^{2}-\frac{1}{n}\times \sum_{i=1}^{n}{\left(p\left(i\right)-p\left(x\right)\right)}^{2}=0. \end{array}$$

The direct consumption coefficient reflects the basic characteristics of the production structure in the Leontief model and is the basis for calculating the complete consumption coefficient. It fully reveals the technical and economic connections between the various sectors of the national economy, that is, the strength of the interdependence and mutual restraint between the sectors, and provides important economic parameters for constructing input-output models.

(3) $$\begin{array}{c} \left\{\begin{array}{c} x\left(i,0\right)=a-x\left(j,0\right),\\ x\left(i,1\right)=b-x\left(j,1\right),\\ x\left(i,j\right)=\sqrt{\frac{x\left(j,i\right)}{a+b}.} \end{array}\right.\\ U\left(x\right)={\left(I-C\right)}^{-1}\times C^{T}-\sum_{i=1}^{n}p\left(x\right)\times C\left(i\right)\sum_{i=1}^{n}p\left(x\right)\times Z\left(i\right). \end{array}$$

Range refers to the difference between the maximum value and the minimum value of a certain index. It reflects the largest absolute difference in the change of a certain indicator among various regions. The range index *g* can indicate the gap between the county with the most developed tourism economy and the county with the least developed tourism economy. The standard deviation is the square root of the square root of the square of the deviation of the standard value of each unit of the population from its mean.

(4) $$\begin{array}{c} g\left(w\left(i\right)|w\left(i-n+1\right),\ldots ,w\left(i-1\right)\right)=\frac{P\left(w\left(i-n+1\right),\ldots ,w\left(i-1\right),w\left(i\right)\right)}{P\left(w\left(i-n+1\right),\ldots ,w\left(i-1\right)\right)}. \end{array}$$

The complete consumption coefficient refers to the sum of the direct and indirect consumption of goods or services in the *i* product sector for each unit provided by the *j* product sector for final use. The complete consumption coefficient of each product department is expressed in the form of a table, which is a complete consumption coefficient table or a complete consumption coefficient matrix, usually represented by the letter *V*.

(5) $$\begin{array}{c} V\left(x\right)=\frac{\sum_{i=1}^{n}\sum_{j=1}^{n}w\left(i,j\right)*\left(x\left(i\right)-x\right)\times \left(x\left(j\right)-x\right)}{\sum_{i=1}^{n}\sum_{j=1}^{n}w\left(i,j\right)\times x\left(i,j\right)}. \end{array}$$

The coefficient of variation is the ratio of the standard deviation to the corresponding average. It can exclude the influence of the difference in units or averages on the comparison of the degree of variation of two or more values. The coefficient of variation *f*(*x*) can explain the relative differences in tourism economy among different research units.

(6) $$\begin{array}{c} \exp\sum_{i=1}^{n}x\left(i\right)f\left(s,t\right)=\exp\;x\left(1\right)f\left(x\right)+\cdots +\exp\;x\left(n\right)f\left(x\right). \end{array}$$

### 2.2. Spatiotemporal Difference Evolution Model

In this article, the difference in the tourism economy based on the regional Internet of Things means that, under the influence of different factors, there are differences in economic levels between different regions in the development of the tourism economy and the unevenness in the development of tourism industry in different regions within a certain period of time.  Figure 2 shows a schematic diagram of the evolution model of temporal and spatial differences. The growth pole refers to a collection of economic units with agglomeration characteristics in space. Economic development will first explode at a certain point in a region and then gradually spread outward from this point, thereby driving the economic development of the entire region. It has a strong economy of scale and it drives the economic development of the entire region through multiplier effects, dominance effects, polarization, and diffusion effects. Some areas developed first to become regional “centers” due to various favorable factors, while other areas became “peripheries” due to lagging development. The center is in a dominant position, while the periphery depends on the center for development, and peripheral funds, materials, and labor will be continuously transferred to the center.

Generally speaking, the lower the level of tourism development is, the lower the consumption level of tourists is, and the higher the proportion of basic tourism consumption expenditure in total consumption expenditure is. At present, as the regional tourism industry is generally in the early stage of development, tourism supporting facilities and services are not yet complete, and the products are single, tourism consumption is mainly used for transportation, accommodation, catering, sightseeing, etc., and the proportion of nonbasic tourism consumption is very small. The change curve of employment elasticity is basically similar to that of the tertiary industry, and the fluctuation range shows a trend of gradual convergence. The employment elasticity of tourism industries showed almost the same changes as the employment elasticity. The purpose of statistical testing is to test the reliability and accuracy of estimated values.  Table 1 shows the statistical test results of tourism characteristic industries. Goodness of fit refers to the degree of fit of the regression line to the observed value. The regression parameter estimation shows that the model fits the sample well.

The tourism characteristic industry belongs to the tertiary industry. There are two main methods for measuring the difference of the tourism economy: relative difference and absolute difference. It shows that the regression equation is significant; that is, the combination of variables such as tourism resource endowment, location and transportation conditions, economic development level, and industrial structure does have a significant impact on the tourism economy. When other variables remain unchanged, the explanatory variables such as the endowment of tourism resources, location and transportation conditions, and the level of economic development have a significant impact on the tourism economy, while the industrial structure has no significant impact on the tourism economy.

### 2.3. The Distribution of Tourism Economic Weighting Factors

The establishment of an indicator system of factors influencing the tourism economy based on the regional Internet of Things requires that the indicators have scientific and clear characteristics and can accurately reflect the main aspects and essential characteristics of factors affecting tourism economy in the county. Based on the correct understanding of the county tourism economy, the influencing factors are classified, and each category corresponds to specific indicators so as to construct the county tourism economy influencing factor index system. Therefore, it is of great significance to develop the tourism industry, to further utilize the potential of tourism characteristic industries to absorb labor, to adjust the regional employment structure, to optimize and upgrade the employment structure, and to achieve the coordinated development of the employment structure and industrial upgrading.

Based on the proximity of counties (cities and districts), the binary adjacency weight matrix is used, and Geoda software is used to calculate the global spatial autocorrelation coefficient of the comprehensive development level of the regional tourism economy. The adjusted goodness of fit was 0.918, indicating that there is a significant linear relationship between the dependent variable and the independent variable. The statistical *t* values are all positive, and the significance level is less than 0.05, indicating that the standard regression coefficient is significant.  Figure 3 shows the two-dimensional scatter point distribution of the goodness of fit of the temporal and spatial differences. Therefore, the equation has a good fitting effect on the whole, indicating that the level of regional economic development can reflect the development of the regional tourism economy to a certain extent. Therefore, when constructing indicators for the comprehensive development level of the tourism economy, this article constructs it from two aspects: tourism industry development level and regional economic development level.

The selected index system needs to be able to scientifically reflect the actual situation of the county tourism economy and faithfully reflect the connotation of the corresponding influencing factors by selecting indicators with strong relevance and high representativeness. The establishment of the index system is ultimately to implement each specific data, so the availability and calculation of the selected index data are required to be strong. Because it is relatively difficult to collect county data, it is necessary to ensure the availability of indicators. The principle of operability is one of the indispensable conditions for establishing a complete index system. The full consumption coefficient refers to the sum of the direct and indirect consumption of goods or services in the *i*-th product sector for each unit provided by the *j*-th product sector for final use. Based on the characteristics of county tourism economy and the principles of influencing factor index system construction, and drawing on some of the latest results of current regional tourism economic research, this article focuses on the four aspects of tourism resource endowment, location and transportation conditions, economic development level, and industrial structure. They are tourism resource endowment, location traffic conditions, economic development level, and industrial structure. Therefore, we can conclude that the endowment of tourism resources affects the tourism economy of the county to a greater extent. The location and traffic conditions are greater than the level of economic development and the industrial structure. This is basically consistent with empirical judgment.

## 3. Results and Analysis

### 3.1. Extraction of Tourism Economic Data

We use SPSS19.0 software to analyze the selected indicators using the orthogonal rotation method with maximum variance. The KMO test result was 0.819, indicating that the principal component analysis method is suitable. Mathematical statistics cannot explore the evolution of economic differences from a spatial perspective. Therefore, this article uses the natural fracture method in ArcGIS software to classify counties and visualize them to analyze the development of the county tourism economy in terms of time. The characteristics of spatial evolution are to make up for the limitations of mathematical statistics in spatial analysis and also reflect the characteristics of geographic research—analyzing the differences in the distribution of things from a spatial perspective. The research needs to use the relevant data of county-level administrative districts.  Table 2 shows the statistics of tourism economic data. This article is to obtain the relevant data in a complete and comprehensive way. By visiting statistical websites of various counties, relevant effective data are collected from statistical yearbooks, statistical reports, or annual national economic and social development reports to reflect the county's tourism economy as comprehensively and accurately as possible.

Through calculations, in the past ten years, the employment scale of the regional tourism industry has shown an overall growth trend, but the volatility is relatively large. The number of employees in the regional tourism industry has reached 961,300, an increase of 24.31% compared to 773,300, and an average annual growth of 2.03%. The proportion of employees in tourism characteristic industries in the total number of employees in the society has increased, from 3.20% to 3.43%, but the proportion of employees in the tertiary industry has declined, from 14.45% to 11.35%. The growth rate of employment is faster than the growth rate of the number of employees in the whole society but obviously lags behind the growth of the number of employees in the tertiary industry. Traditional labor-intensive industries such as the postal industry have become the main industries for absorbing labor in the tertiary industry in the region, with an employment ratio of more than 10%. It can be seen that the selected index data reflecting the level of regional tourism economic development have been subjected to principal component analysis and dimensionality reduction, and four principal components have been extracted. The characteristic value of principal component one is 5.665, and its principal component contribution rate is 47.206%. The characteristic value of principal component two is 1.737, and its principal component contribution rate is 14.472%. The characteristic value of principal component three is 1.319, and its principal component contribution rate is 10.992%. The characteristic value of principal component four is 1.178, and its principal component contribution rate is 9.819%. Its cumulative variance contribution rate has reached 8.489%.  Figure 4 shows the statistical distribution of the contribution rate of tourism economic variance. The eigenvalues of the four principal components are all greater than 1, indicating that the extracted four principal components can well describe the comprehensive difference of tourism economic differences.

We use multiple linear regression to analyze the correlation between tourism economic development level and tourism resource endowment, location traffic conditions, economic development level, industrial structure, and other factors and judge the degree of influence of different factors on dependent variables. From the analysis of the causality test results of the two variable combinations composed of each influencing variable and the employment elasticity of tourism characteristic industries, there is a certain one-way relationship between labor factors and the employment elasticity of tourism characteristic industries. Both the differences between prefectures and cities and the differences within prefectures and cities show a downward trend in fluctuations. The decline from 0.934 to 0.469 shows that the regional differences in total tourism revenues within cities are gradually decreasing.

## 4. Simulation of Temporal and Spatial Difference Evolution Model

In order to further comprehensively study the regional differences in regional tourism, this article extracts *X*1 domestic tourism income, *X*2 tourism foreign exchange income, *X*3 domestic tourists, and *X*4 international tourists. As an explanatory variable of the effect of regional tourism employment, it is not only necessary to analyze it from the scale of employment but also to grasp it from the quality of employment. Therefore, the absolute amount of tourism employment and the elasticity of tourism employment are selected for measurement. Here, GH, TH, GT, and TT are used to denote the employment scale of tourism core industry, the employment elasticity of tourism core industry, the employment scale of tourism characteristic industries, and the employment elasticity of tourism characteristic industries. Such a statistical caliber is obviously not enough to reflect the actual situation and overall picture of the tourism industry, and it cannot reflect the corresponding status and role of the tourism industry in the national economy.  Figure 5 shows a line chart of the proportion of the tourism economy in the total value. This article uses international and domestic tourist visits (TP) and international and domestic tourism revenue (TC) to characterize tourism demand factors, selects fixed asset investment (FAI) and tourism institutions (TS) in industries that are highly related to tourism economic growth to characterize tourism supply factors, and uses gross domestic product (GDP), the proportion of tertiary industry gross product (TIG), and per capita income (PCI) to characterize economic environmental factors.

It is difficult to select appropriate variables for the influencing factors of county tourism spatial differences. In order to better measure each influencing factor, it is necessary to rationally sort and process the original data. This article has made many adjustments to the selection of data through multiple calculations of SPSS. The contribution index of the county tourism economy to the national economy is the proportion of the county's total tourism revenue to the regional GDP. According to the calculation results, the county tourism industry with a contribution index between 0 and 0.10 is named a general industry, the county tourism industry with a contribution index between 0.10 and 0.20 (including 0.10) is named as a pillar industry, and the county-level tourism industry with a contribution index between 0.20 and 0.30 (including 0.20) is named an important pillar industry, and the contribution index is at 0.20. County tourism industries above 30 (including 0.30) are named as strategic pillar industries.  Figure 6 shows a fan chart based on the contribution index of the regional Internet of Things. And through ArcGIS software, these four levels of counties are presented in different colors to analyze the spatiotemporal evolution analysis of the difference in the contribution of the county tourism economy to the national economy. The total tourism income of the counties (cities and districts) in the district is extremely poor, and the standard deviation is increasing. The coefficient of variation and Theil coefficient show a downward trend in fluctuations, indicating the absolute value of the total tourism income of the counties (cities and districts) in the district. The difference shows an accelerated growth trend, and the relative difference in total tourism revenue is gradually shrinking.

We divide the total swimming rate into three levels: in the first level, the total swimming rate is extremely low, which is less than 100%; in the second level, the total swimming rate is low, which is 100% to 200%; and in the third level, the general swimming rate is high, which is between 200% and 300%. We can see that the travel rate anomalies of the cities and states in the region are obvious differences in the value. In some areas, the anomaly values are positive and some are negative. According to the data, we divide the total travel rate anomalies of each city and state into three categories: in the first category, the total travel rate has an anomaly value greater than 50%; the second category refers to areas where the total travel rate is close to the average level, and the total travel rate anomaly is lower than 50%; and the third category refers to areas with a large proportion of total employment in tourism, tourism is also the main area for absorbing labor in the region, accounting for a large proportion of total employment in the region, and the proportions of the cities and districts are basically the same. The inbound travel rate anomaly is divided into two categories: the first category is the inbound travel rate level and the second category is areas where the inbound travel rate is lower than the average level, and the anomaly value is negative. The global index of the total tourism revenue of each county (city and district) in the region is positive and shows a trend of increasing in fluctuation, indicating that there is a significant spatial correlation in total tourism revenue.

### 4.1. Example Application and Analysis

We divide the inbound travel rate into four levels. The first level refers to areas with an inbound travel rate of less than 0.1%, the second level refers to areas with an inbound travel rate of 0.1% to 1%, the third level refers to areas where the inbound travel rate is between 1% and 2%, and the fourth level refers to areas where the inbound travel rate is greater than 2%. By comparing the number of tourism employment driven by unit income, it reflects the contribution of tourism to the employment of various regions and cities in the region and at the same time measures the imbalance in the development of this indicator between regions. Its size depends on the growth rate of the tourism economy and labor productivity. From a spatial comparison, the better the economic foundation is and the stronger the comprehensive strength of tourism economy development is, the smaller the number of jobs driven by tourism income is, basically between 0.10 and 0.15. Both the extreme value ratio and the coefficient of variation show an obvious growth trend, which can be seen intuitively.  Figure 7 shows the histogram of the average annual growth rate of the tourism economy. From the comparison of the number of tourism employment driven by tourism income, the tertiary industry GDP, and the unit income of the regional GDP, the number of employment driven by tourism income per labor is the smallest. These reflect that, from the perspective of industry comparison, the output level of unit tourism labor is relatively high; from the perspective of prefecture and city comparison, the tourism labor productivity of economically developed regions is relatively high. In other words, the tourism economy of underdeveloped regions has a relatively high strong labor-absorptive capacity.

Counties with a ranking improvement of more than 10 places are named rapid development type, and counties with a ranking improvement between 0 and 10 places (including 0 and 10) are named development type, and counties with ranking regressed by 1 to 10 places (including 10) are named lagging type, and counties with ranking regressed by more than 10 places are named significantly lagging type. And we use ArcGIS software to make a spatial visualization map to explore the law of spatial change. The scale of fixed asset investment in the region has shown the characteristics of continuous increase, with an average annual growth rate of 18.25%, which is nearly 5 percentage points higher than GDP. The contribution rate of fixed asset investment to economic growth has reached 58.40%, which has risen to around 70% in recent years. Fixed asset investment has the dual function of regulating supply and demand. The long-term growth of accumulation and investment is the most basic condition for a large amount of surplus labor to be absorbed by the economy. On the one hand, continuous large-scale investment balances the original labor and capital. The relationship is broken, which promotes employment growth; on the other hand, it indirectly drives the expansion of investment and employment in other related sectors through the multiplier effect. The range increased from 149.54 to 718.83, and the average annual growth rate reached 20.4%. And in recent years, the growth has been particularly obvious, and the range has grown rapidly from 483.87 to 718.83, a growth rate of 48.56%. The growth of the standard deviation is very similar to that of the extreme deviation, but the growth rate is faster.  Figure 8 shows a line chart of the growth rate of the tourism economy.

Through the analysis of the correlation between regional tourism employment effect variables and various influencing factors, it can basically be judged that the employment scale of core tourism industries and characteristic industries has a strong same-directional relationship with various influencing factors, and the significance level is obvious. The employment elasticity of characteristic industries has a weak and inverse relationship with various influencing factors, and its significance level is not obvious. It can be found that regional tourism can have an impact on almost all industrial sectors in terms of employment, but the employment effects of different industrial sectors are affected by tourism. The focus of this method is to explore the distribution of spatial data, so it is necessary to measure the correlation coefficient between the data. According to a comprehensive analysis, the accommodation and catering industries are most affected. The comprehensive employment coefficient of each tourism characteristic industry is 2.0015, that is, every characteristic industry gains 10,000 yuan of added value, which can lead to 20,015 employment opportunities in the accommodation and catering industry. This is followed by the manufacturing industry at 1.9477 and the tourism core industry at 1.4686.

## 5. Conclusion

This paper analyzes the statistical data of tourism economy based on the regional Internet of Things and concludes that the absolute difference in the unbalanced development of the county tourism economy is expanding, the relative difference is constantly shrinking, and the degree of concentration of the county tourism economy is decreasing, and it is developing in a balanced direction. This article analyzes the temporal and spatial evolution characteristics of county tourism economic differences from three aspects: the difference in the total county tourism income, the difference in the contribution of the county tourism economy to the national economy, and the difference in the ranking changes of the county tourism economy in the province. This paper follows the structural model of the tourism development dynamic system, combines the theoretical ideas of employment growth, considers the unique attributes of the tourism industry, and establishes an interactive type composed of tourism demand and tourism element supply and connected by the economic environment and labor conditions. The focus of this method is to explore the distribution law of spatial data, so it is necessary to measure the correlation coefficient between the data to determine whether the data has a spatial relationship and the strength of the relationship. From the spatial dimension, we take the regional city as the basic research unit, take the number of employment in tourism characteristic industries as the research caliber, adopt multiple indicators, and conduct a comprehensive evaluation of the regional development of regional tourism employment through horizontal and vertical comparisons. We use SPSS19.0 to establish a multiple linear regression model of important factors affecting regional tourism economy to analyze the factors affecting regional tourism economic differences. Finally, the countermeasures and suggestions for promoting the sustainable development of the regional tourism economy are put forward, with a view to narrowing the difference of the regional tourism economy and promoting the coordinated development of the tourism economy.

## Figures and Tables

**Figure 1:** Spatial nesting of regional IoT.

**Figure 2:** Schematic diagram of the evolution model of temporal and spatial differences.

**Figure 3:** Two-dimensional scatter point distribution of goodness of fit of temporal and spatial differences.

**Figure 4:** The statistical distribution of the contribution rate of tourism economy variance.

**Figure 5:** Line chart of the proportion of tourism economy in the total value.

**Figure 6:** Fan chart of contribution index based on regional IoT.

**Figure 7:** Histogram of average annual growth rate of tourism economy.

**Figure 8:** Line chart of growth rate of tourism economy scale.

**Table 1:** Statistical test results of tourism characteristic industries.

Unit index	Coefficient of elasticity	Goodness of fit	Return parameters
1	0.03	0.97	1.44
2	0.07	0.96	3.71
3	0.05	0.89	2.36
4	0.08	0.87	2.53

**Table 2:** Tourism economic data statistics.

Area code	Employed population (×10^4^)	Growth rate (%)	Variance contribution rate (%)
1	91.13	22.13	37.56
2	64.71	18.52	39.07
3	82.02	19.17	18.84
4	77.52	26.03	24.57
5	79.72	9.42	47.06

## Data Availability

The data used to support the findings of this study are available from the corresponding author upon request.
